# Consequences of hydrogenated vegetable fat substitution with Ajwa seed oil on physicochemical and nutritional aspects of functional cookies

This article has been retracted.

**DOI:** 10.1002/fsn3.1383

**Published:** 2020-02-03

**Authors:** Muhammad Qasim Raza, Muhammad Umair Arshad, Muhammad Sajid Arshad, Faqir Muhammad Anjum, Ali Imran, Aftab Ahmed, Haroon Munir

**Affiliations:** ^1^ Institute of Home and Food Sciences Government College University Faisalabad Pakistan; ^2^ Vice Chancellor University of The Gambia (UTG) Banjul Gambia

**Keywords:** Ajwa date seed oil, antioxidant activity, cookies preparation, functionality, hydrogenated vegetable fat, palatability

## Abstract

The core objectives of the current study were to explore and compare the proximate and nutritive composition of both types of cookies prepared either with Ajwa seed oil (ASO) or hydrogenated vegetable fat (HVF) and comparative analysis of the antioxidantal potential of both cookies and to reconnoiter the storage effects on the quality parameters of the cookies over a period of 60 days. Outcomes revealed that the cookies prepared with the ASO were superior (*p* < .05) in fat% and energy as compared to the cookies with HVF. Due to the presence of functional moieties, ASO cookies were found with better palatability, increased shelf life with enhanced physical properties and better functionality. Therefore, the findings of the current study revealed that ASO could be used as an alternative fat source for the preparation of novel functional cookies instead of conventional vegetable fats.

## 1 INTRODUCTION

Date (*Phoenix dactylifera* L.) is believed to be the hoariest food produce being consumed by the mankind for more than 6,000 years (Kwaasi, 2003), included in the family *Palmae,* and is under cultivation across the globe because of its popularity among the masses and its wide acceptability to an extensive range of ecological regions including arid to semiarid regions (Al‐Farsi & Lee, 2008). Date seed being the discarding material with the availability of very limited information about its viability used as an active ingredient for the preparation of functional foods except for its utilization in animal feed after its separation from the date fruit and is supposed to be very rich in bioactive constituents as evident from the outcomes of various studies (Aldhaheri, Alhadrami, Aboalnaga, Wasfi, & Elridi, 2004; Besbes et al., 2005).

Dietary guidelines are relaying with great concern upon the health‐promoting characteristics of phytochemicals as they impart proven beneficial impacts on human health against different diseases including cardiovascular disease (CVD), diabetes, obesity, and neurodegenerative complications (Jayasekera, Molan, Garg, & Moughan, 2011). There are different date cultivars having different health benefits. Ajwa dates have better cholesterol‐lowering potential and antiobesity effect than number of other cultivars (Arshad et al., 2019). In order to curtail different disorders and ailments, the effectiveness of phytochemicals has inspired its supplementation especially from plant‐based nutraceuticals because of their diversity and availability (Xin, Yuan, Xiao, & You‐Ying, 2011). Plant‐based intrusions are dependent on their active constituents commonly known as the plant secondary metabolites, and these compounds are most widely dispersed in plant kingdom including phenolics in their different forms including carotenoids, flavonoids, sterols, lignins, and tannins (Blainski, Lopes, & De Mello, 2013). Currently, people are more concerned and interested in nutritious and diet‐based treatments especially from vegetative sources; in turn, food industries are starving for such plant‐based functional and nutraceutical foods that can fulfill the self‐esteems of their target groups (Jisha, Padmaja, Moorthy, & Sajeev, 2009). Further due to the sedentary life styles of the communities, demand for ready to eat packaged food products is increased that in turn demands an overall improvement of the quality parameters (Nanditha & Prabhasankar, 2009).

Fats are the key energy source and an imperative constituent of a healthy diet that is responsible for improving the taste, aroma, and texture of the food products along with a positive neurological stimulus of fullness after its ingestion in addition to carbohydrates and proteins (Alfenas & Mattes, 2003). Excess of reactive oxygen species (ROS) which interact as free radicals of oxygen resulted from oxidative stress, and in order to combat these harmful effects, it is very important to supplement the body with micronutrients from external sources especially from oil containing foods enriched with antioxidants that can easily overcome the problem of unwanted progression of oxidation that ultimately results in rancidity (Aslam et al., 2018). Value addition of waste or discarding material is cost‐effective while improving the shelf life of the products needs extra cost (Reddy, Urooj, & Kumar, 2005). Therefore, it is believed that partially hydrogenated vegetable fats (HVF) are the richest source of trans‐fats being carcinogenic and supposed to be unhealthy, and need to be replaced with some healthy alternatives without affecting the quality parameters and sensory attributes (Wang, Gravelle, Blake, & Marangoni, 2016).

Ajwa date seed oil (ASO) is characterized by its defensive properties due to its excellent antioxidant status that is helpful against treatment of different metabolic syndromes in addition to its antidiabetic, antimicrobial, anti‐inflammatory, nephroprotective activities and helping in delivery and labor relaxation (Arshad et al., 2014).

Ajwa seed oil (ASO) is believed to be very stable against oxidation because of having an ample quantity of natural antioxidants including flavonoids and nonflavonoids, such as rutin, catechin, and caffeic acid (Besbes et al., 2005; Hamad et al., 2015). Ajwa seeds are known to have a potential of 8%–10% of oil which is regarded as oleic–linoleic oil. Hence, Ajwa date oil on characterization showed very good quality indicators of acid value (AV) being 1.5 mg KOH/g and iodine value (IV) of 59.9 g I_2_/100 g. The free fatty acid (FFA) percentage is about 3.1%, saturated fatty acids (SFAs) amounting about 21.2%, and mainly comprised of palmitic acid (10.3%), myristic acid (5.6%), lauric acid (3.2%), and steric acid (2.1%), whereas unsaturated fatty acids (USFAs) constitutes about 75.26% of ASO comprising mainly oleic acid (66.1%), linoleic acid (8.3%), and linolenic acid (0.86%) (Galeb et al., 2012).

In product development, very limited information is available which could elucidate the use of date seed oil (DSO) in the making of novel functional recipes for human consumption except in concocting mayonnaise, where utilization of DSO as a substitute to corn fat is evident (Basuny & Al‐Marzooq, 2011). Further, the use of dietary fiber from Ajwa date seeds in bakery products is evident from the outcomes of a number of studies suggested that this potential of the dietary fiber could be utilized for their health benefits (Rahman, Kasapis, Al‐Kharusi, Al‐Marhubi, & Khan, 2007). Additionally, it is evident from the previous studies that date seeds have excellent constituents including its oil that could have a diverse acceptability in the pharmaceutical and cosmetic industry. With a strong recommendation to explore, its health and beneficial aspects further by its incorporation in the development of functional food products for human consumption with an insight to curtail the various complications and disorders (Devshony, Eteshola, & Shani, 1992). It is acceptable that replacing the conventional vegetable fats being unhealthy for the preparation of cookies with ASO could impart positive attributes of quality and functionality in addition to the improved health claims (Besbes, Blecker, Deroanne, Bahloul, et al., 2004; Besbes, Blecker, Deroanne, Drira, & Attia, 2004). Further, substitution of animal fats especially butter with an emulsion of oils resulted in overall improved health claims and consumer convenience (Giarnetti, Paradiso, Caponio, Summo, & Pasqualone, 2015).

## 2 MATERIALS AND METHODS

### 2.1 Materials

Two different types of cookies were prepared according to the method of AACC (2000) with trivial changes of substitution of fat type, temperature, and baking time. First type of cookie was prepared with conventional HVFs or shortenings containing a blend of palm oil, canola oil, and soybean oil 100%. While in second type of cookie, 100% ASO was used instead of HVF or plastic fats. All the ingredients used in accordance with a specified recipe were procured locally, and then were weighed and utilized further. All the ingredients other than ASO were in the following proportion fine flour or cake (40%), whole meal flour (15%), eggs (5%), salt (0.40%), sugar (2.0%), NaHCO_3_ (5%), and almond extract (0.05%). While the source of fat for the both types of cookies were including ASO extracted directly from Ajwa date seeds at a rate of 33% for ASO cookies and HVF or shortenings a blend of canola, palm, and soybean oil at a rate of 33% for HVF cookies. Ajwa seed oil was extracted by following the protocol of Mortadha, Tahseen, and Imad (2015) in accordance with AOAC (1990) through solvent extraction method and was used further.

All the ingredients as per standard recipe were mixed thoroughly in a two‐step mixing process. At first step, all the dry ingredients were mixed at a lower speed of mixer for a time of approximately 2 min followed by addition of eggs and then the addition of fat source either ASO or HVF in small proportion to the dry ingredients under mixing to facilitate the through mixing. In the second stage, the remaining fat source (ASO or HVF) was added and the speed of the mixer was increased up to 60 rpm for a time of 10 min. The whole mixing process was completed in approximately 15 min, and at the end, almond extract was added followed by sheeting of cookies in 12–15 g aliquots for the preparation of 900–950 cookies. Two batches of cookies, one with ASO and other with HVF, were prepared each of 15 kg in a commercial baking oven at a temperature of 175°C for 15–20 min. Cookies with golden color that was the indication of proper baking were obtained and allowed to cool and weighed individually. Cookies were then placed in airtight food grade glass containers at ambient room temperature (25 ± 5°C) for a period of 60 days. There were a total of 12 airtight glass containers, 6 each with ASO and HVF cookies, and each glass container was consisted of 160–170 cookies of each type. One container of each type of cookie (ASO and HVF) was opened, and the cookies were analyzed at each data collection period (baseline, 30th, and 60th days).

### 2.2 Methods

#### 2.2.1 Proximate analysis

Functional cookies were analyzed for following attributes during 60 days of storage at baseline, 30th and 60th days. Proximate analyses were carried out by following the standard methods as described in AACC (2000), including determination of crude fat (CF) by method No. 30‐25, moisture contents (MC) through method No. 44‐15A, crude protein (CP) meant by method No. 46‐30, crude fiber (Cf) against method No. 32‐10, and ash contents (AC) from method No. 08‐01.

#### 2.2.2 Moisture contents (MC)

Moisture was determined by using an air‐dried oven (Blodgett; CTB/CTBR) by following the standard protocol No. 44‐15A (AACC, 2000). The percent (%) of moisture was estimated from the expression given below:

$$\text{Moisture}\;\left(\%\right)=\frac{W_{1}}{W_{2}}\times 100.$$

#### 2.2.3 Crude protein (CP)

Percentage of CP was estimated by using Kjeldahl's apparatus method No. 46‐13 (AACC, 2000). CP in percent (%) was measured by multiplying nitrogen (N) with a factor of 5.70.

#### 2.2.4 Crude fat (CF)

CF (%) content was evaluated by means of Soxhlet extractor using n‐hexane as solvent for at least 04 hr by taking 5 g sample following the standard protocol No. 30‐25 (AACC, 2000). The % of CF was estimated from the expression given below:

$$\text{Fat}\;\left(\%\right)=\frac{\left(\text{weight of fat}\right)}{\left(\text{weight of sample}\right)}\times 100.$$

#### 2.2.5 Crude fiber (Cf)

The Cf content was determined using the standard protocols No. 32‐10 (AACC, 2000). Crude fiber content was estimated by using muffle furnace (Thermo scientific Thermolyne F48010‐33). The % of Cf was estimated from the expression given below:

$$\text{Fiber}\;\left(\%\right)=\frac{\left(\text{weight loss}\right)}{\left(\text{weight of sample}\right)}\times 100.$$

#### 2.2.6 Ash contents

Ash was determined by following method No. 08‐01 AACC (2000), by means of an electric muffle furnace through incineration at high temperature (Thermo scientific Thermolyne F48010‐33). The % of ash content was estimated from the expression given below:

$$\text{Ash}\;\left(\%\right)=\frac{A-B}{C}\times 100.$$

#### 2.2.7 Antioxidant potential

Antioxidant potential was estimated by calculating peroxide value (PV), acid value (AV), energy, nitrogen free extract (NFE), and thiobarbituric acid (TBA) value following the standard protocols of AACC (2000). Furthermore, total rutin, catechin, and caffeic acid of the cookies were assessed following the method of Lunn (2000).

#### 2.2.8 Peroxide value (POV)

Firstly, ash contents were estimated through AACC (2000). In order to remove the impurities, the sample was ignited and filtrated through filter paper. Under the same conditions, a blank reading was also obtained. The POV was quantified through the following expression:

$$\text{Peroxide Value}=\frac{(B-A)\times N\times 1000}{W}$$

where *B* = Vol. of Na_2_S_2_O_3_ used for blank, *A* = Vol. of Na_2_S_2_O_3_ used for sample, *N* = Normality of Na_2_S_2_O_3_, *W* = Weight of oil taken.

#### 2.2.9 Total acidity (AV)

AV was estimated by following the standard protocol of AACC (2000). AV was determined by following the given expression:

Acid Value=56.1VN.

#### 2.2.10 Nitrogen free extract (NFE)

The nitrogen free extract was quantified from the given equation:

NFE%=100-(Moisture%+Ash%+Fat%+Fiber%+Protein%)

#### 2.2.11 Thiobarbituric acid value (TBA)

Assessment of lipid oxidation was measured by evaluating the development of TBARS by adopting the protocol as narrated by Garcia‐Alonso, De Pascual‐Teresa, Santos‐Buelga, and Rivas‐Gonzalo (2004) with trivial changes. A blank sample was heated for 35 min in a water bath in the presence of TBA reagent, and then, it was allowed to cool for 10 min in water and absorbance (D) against the blank sample was measured at 538 nm wavelength by spectrophotometer following the standard protocol of AACC (2000).

TBA no. was estimated by the following equation:

$$\text{TBA No}.\;\left(\text{mg malanaldehyde per kg sample}\right)=7.8\times$$

#### 2.2.12 Active ingredient determination

Both types of cookies were analyzed for total rutin, catechin, and caffeic acid following the method of Lunn (2000) with slight changes. About 2 g of ASO or HVF cookies sample was taken in a test tube, 20 ml methanol was added, and then, it was allowed to vortex for half an hour. Then, the sample was centrifuged at 2,500 rpm for another half an hour. Upper layer of the centrifuged was isolated, and the remaining sample was extracted against the methanol solution followed by combining the both extractions and further evaporation in the presence of nitrogen. This evaporated sample was then added with 2 ml of methanol solution followed by vortex. Prepared sample was then injected in HPLC with a mobile phase of methanol and water (70:30v/v) at a flow rate of 1 ml/m equipped with C_18_ column (4.6 mm × 150 mm), and the UV was adjusted at 288 nm. Rutin, catechin, and caffeic acid were estimated by comparing with their respective standards.

#### 2.2.13 Physical properties and palatability

Palatability of the both types of cookies was evaluated by means of sensory evaluation following the protocol of Meilgaard, Civille, and Carr (2007). For sensory evaluation, an accessible heterogeneous population of different age groups comprised of 100 people including males and females from academia and general public were engaged for all three times evaluation. It was noted that 75 people out of 100 participated in all three times evaluation. Participants were provided with both types of cookies at each time in precoded cups, and every participant was asked to taste 3 cookies of each type at each time for evaluation on 9‐point hedonic scale, and mineral water was given to neutralize the taste after every single evaluation by following the protocol of Meilgaard et al. (2007). The physical characteristics were also determined by the panelists at all three times by using three cookies from both groups including diameter and size of cookies in addition to their thickness and spread factor (AACC, 2000).

#### 2.2.14 Statistical analyses

For proximate analysis and physical characteristics, all data were obtained in triplicate and were expressed as mean ± *SE*; for the palatability attributes, the data obtained from the participants at all three times were evaluated. Two‐way ANOVA was applied to the all data obtained with a value of *p* ≤ .05 was expressed as highly significant (Steel, Torrie, & Dickey, 1997).

## 3 RESULTS AND DISCUSSIONS

### 3.1 Physicochemical analysis of cookies

Physicochemical analyses of both types of cookies are presented in Table 1 over a period of 60 days. Ajwa seed oil cookies were prepared with 100% ASO, while the HVF cookies were prepared with 100% HVF or shortenings a blend of palm, canola, and soybean oil. At baseline, the moisture content in ASO cookies was 2.68 ± 0.01%, while the MC in HVF cookies was found as 2.60 ± 0.01%. Further, the crude fiber contents at baseline in ASO cookies were 2.15 ± 0.01% and HVS cookies were 2.09 ± 0.01%. Similarly, the ash contents in ASO and HVS cookies at baseline were 0.940 ± 0.010% and 0.903 ± 0.015%, respectively. At baseline, ASO cookies had significantly (*p* < .05) higher protein contents 8.23 ± 0.01% as compared with the HVS cookies 7.83 ± 0.00%. At the termination of the storage study, the MC of ASO cookies increased from 2.68 ± 0.01% at baseline to 3.56 ± 0.02% at 60th day of storage, whereas the moisture contents of HVF cookies also found significantly (*p* < .05) increased from 2.60 ± 0.01% at baseline to 3.72 ± 0.02% at 60th day, while protein, fat, fiber, and ash contents significantly decreased in ASO cookies from baseline to 60th day of storage as 8.23 ± 0.01% to 8.03 ± 0.03%, 39.61 ± 0.01% to 38.41 ± 0.01%, 2.15 ± 0.01% to 2.00 ± 0.01%, and 0.940 ± 0.010% to 0.900 ± 0.010%, respectively. On the other hand, moisture contents in HVF cookies increased from 2.60 ± 0.01% at baseline to 3.72 ± 0.02% at 60th day. Similarly, crude protein, crude fat, crude fiber, and ash contents were decreased in HVF cookies from baseline to 60th day of storage. Moisture contents were significantly (*p* < .05) higher in HVF cookies, while rest of the constituents were lesser in HVF cookies as compared with ASO cookies.

**Table 1:** Proximate composition of functional cookies made from Ajwa seed oil

Components	Day 0	Day 30	Day 60
Moisture (%)			
ASO	2.68 ± 0.01e	3.33 ± 0.02c	3.56 ± 0.02b
HVF	2.60 ± 0.01f	3.20 ± 0.01d	3.72 ± 0.02a
Protein (%)			
ASO	8.23 ± 0.01a	8.16 ± 0.01b	8.03 ± 0.03c
HVF	7.83 ± 0.00d	7.71 ± 0.02e	7.56 ± 0.01f
Fat (%)			
ASO	39.61 ± 0.01a	38.81 ± 0.01b	38.41 ± 0.01c
HVF	36.74 ± 0.02d	35.89 ± 0.01e	35.46 ± 0.02f
Fiber (%)			
ASO	2.15 ± 0.01a	2.07 ± 0.01b	2.00 ± 0.01c
HVF	2.09 ± 0.01b	2.00 ± 0.01c	1.98 ± 0.02d
Ash (%)			
ASO	0.940 ± 0.010a	0.920 ± 0.010ab	0.900 ± 0.010b
HVF	0.903 ± 0.015b	0.833 ± 0.029c	0.763 ± 0.012d
NFE (%)			
ASO	46.39 ± 0.03f	46.72 ± 0.02e	47.08 ± 0.06d
HVF	49.84 ± 0.03c	50.37 ± 0.03b	50.51 ± 0.02a

Note

Means showing similar letter(s) in a row/column are nonsignificant (*p* > .05, *n* = 3). Mean ± *SE*.

Upsurge of moisture contents in cookies during storage over a period of time is evident from the outcomes of Nagi, Kaur, Dar, and Sharma (2012). An increase in MC is responsible for an escalation of various parameters of antioxidant potential determinants including POV, AV, TBA, and NFE that in turn affect the shelf life of the product during storage which is directly proportional to the hygroscopic nature of the dry ingredients. On the other hand, an increase in the moisture content results in a noticeable decrease of proximate constituents including CP, CF, crude fiber, and ash contents mainly responsible for absorbance of excessive moisture contents, and their removal is responsible for an upsurge in MC. Effects and after effects of decreasing and increasing of ash contents on the increase and decrease of moisture are evident from the studies conducted by Waheed, Rasool, and Asghar (2010) and Pasha, Butt, Anjum, and Shehzadi (2002). When compared with other vegetable oils, ASO being oleic–linoleic in nature is enriched with saturated (21.2%) and unsaturated (75.26%) fatty acids. Ajwa seed oil being good source of oleic acid and lower in linoleic acid contents could be compared with the oleic and linoleic acid contents of canola oil, other commercially available vegetable oils and rice bran oil (Abdul Afiq, Abdul Rahman, Che Man, Al‐Kahtani, & Mansor, 2013). On characterization, date seed oil is considered to be oleic and lauric oil (Biglar et al., 2012; Devshony et al., 1992) as compared with coconut and palm oil that is regarded as lauric–myristic and palmitic–oleic oils correspondingly (Devshony et al., 1992). Different studies elucidate that vegetable oils from plant origin are rich in functional moieties that in turn improve the functionality and shelf life of the product; therefore, the replacement of conventional plastic fats or shortenings with vegetable oils could impart positive heath impacts in addition to improved physical properties and palatability (Sharif et al., 2003).

### 3.2 Antioxidant potential of cookies

Table 2 reveals about the antioxidant potential of both ASO and HVF cookies from baseline to the 60th day of storage period. POV of ASO cookies increased from 0.146 ± 0.003 meq/kg at baseline to 0.481 ± 0.001 meq/kg at 60th day; similarly, POV of HVF cookies increased from 0.197 ± 0.002 meq/kg at baseline to 0.531 ± 0.001 meq/kg at 60th day. Acid value of both types of cookies increased from baseline to the 60th day and TBA value in ASO and HVF cookies increased from baseline 0.051 ± 0.002 mg M/kg to 0.074 ± 0.002 mg M/kg at 60th day and 0.062 ± 0.002 mg M/kg to 0.089 ± 0.001 mg M/kg, respectively. Bioactive constituents of flavonoids and nonflavonoids were present in ASO cookies but the same was absent in HVF cookies. Rutin contents were decreased significantly (*p* < .05) in ASO cookies from 6.95 ± 0.01 mg/kg at baseline to 6.75 ± 0.01 mg/kg at day 60; further, catechin contents in ASO cookies also decreased significantly (*p* < .05) over time, and same pattern of significant (*p* < .05) decrease was observed in case of caffeic acid in ASO cookies from baseline 7.80 ± 0.02 mg/kg to day 60 7.71 ± 0.01 mg/kg. There were no bioactive components detected in HVF cookies.

**Table 2:** Antioxidant potential of functional cookies made from Ajwa seed oil

Treatment	Day 0	Day 30	Day 60
POV (meq/kg)			
ASO	0.146 ± 0.003f	0.351 ± 0.001d	0.481 ± 0.001b
HVF	0.197 ± 0.002e	0.440 ± 0.001c	0.531 ± 0.001a
AV (%)			
ASO	0.158 ± 0.000f	0.188 ± 0.001d	0.197 ± 0.001c
HVF	0.183 ± 0.001e	0.199 ± 0.001b	0.218 ± 0.001a
TBA (mg M/kg)			
ASO	0.051 ± 0.002f	0.070 ± 0.002c	0.074 ± 0.002b
HVF	0.062 ± 0.002e	0.066 ± 0.002d	0.089 ± 0.001a
Rutin (mg/kg)			
ASO	6.95 ± 0.01a	6.77 ± 0.01b	6.75 ± 0.01c
HVF	0.00 ± 0.00d	0.00 ± 0.00d	0.00 ± 0.00d
Catechin (mg/kg)			
ASO	8.49 ± 0.01a	8.41 ± 0.01b	8.39 ± 0.01c
HVF	0.00 ± 0.00d	0.00 ± 0.00d	0.00 ± 0.00d
Caffeic acid (mg/kg)			
ASO	7.80 ± 0.02a	7.75 ± 0.01b	7.71 ± 0.01c
HVF	0.00 ± 0.00d	0.00 ± 0.00d	0.00 ± 0.00d

Note

Means showing similar letter(s) in a row/column are nonsignificant (*p* > .05, *n* = 3). Mean ± *SE*.

Ajwa seed oil being self‐sufficient in antioxidants, especially the polyphenols including flavonoids and nonflavonoid bioactive components (i.e., rutin, catechin, and caffeic acid) which in turn make the ASO highly stable against the thermal stress of high temperature (160–250°C) and the concentration of these functional moieties almost remain the same during storage with a, neglected decreasing trend over long storage periods (Sumaira, Nauman, Rao Sanaullah, Haroon, & Asif, 2017). Similarly, Guizani, Suresh, and Rahman (2014) premeditated the thermal properties of different date seed oils and their functional constituents and found two types of peaks in their differential scanning calorimetry (DSC) thermogram, where 1st peak was observed due to the melting of date seed oil and a 2nd peak was visible due to the melting of solids called endothermic peaks; further, they concluded that the melting enthalpy was found in an increased manner while the temperature of the melting peak was found in a deceasing sequence and this temperature increased rapidly with an elevated rate of heating. When talking about the improvement in nutritional aspects of cookies, it means that none of the ingredients were increased in quantity but it denotes that the cookies prepared with ASO were stable enough against the drastic effects of oxidative stress during storage period due to the self‐sufficiency of ASO in bioactive constituents. Furthermore, the storage material also plays a vital role in the desired quality of the final product over a storage period and a number of studies in this domain claim that the physicochemical, antioxidantal potential, and acceptability of the cookies is highly affected by the storage material especially polythene during storage (Rangrej, Shah, Patel, & Ganorkar, 2015). Moisture contents and antioxidantal potential are indirectly proportional to each other means on increasing moisture contents antioxidantal potential decreased. Since the increasing trend of moisture contents was observed in both types of cookies, that is, ASO and HVF cookies, it was observed that ASO cookies were more stable than HVF cookies due to the presence of functional moieties in sufficient quantities as compared with HVF cookies that were found deficient in antioxidant constituents. A number of studies showed that antioxidants exhibit the key role in the improved shelf life and stability of the bakery products (Nanditha & Prabhasankar, 2009). Results of the study conducted by Sharif et al. (2003) showed that the cookies prepared with the vegetable oils having ample quantities of functional contents, that is polyphenols, were superior in the quality parameters, functional characteristics, sensorial attributes, and acceptability of the final product with improved shelf life and healthful effects. Findings of the current investigation are in close agreement with that of Quilez, Ruiz, Brufau, and Rafecas (2006) and Reddy et al. (2005) concluded that using Ajwa date seed oil in the preparation of novel functional food products especially cookies having noticeable quantities of antioxidants especially phenolic acids are responsible for the overall improved quality and enhanced stability of the cookies throughout the storage period of 60 days.

### 3.3 HPLC phenolic quantification

Mean values of phenolic compounds in both types of cookies are evident from Table 2. The HPLC analysis showed that ASO based cookies contained 6.95 ± 0.01 mg/kg of rutin at baseline to 6.77 ± 0.01 mg/kg on 30th day and 6.75 ± 0.01 mg/kg on 60th day of storage, while rutin contents in the cookies prepared with HVF on analysis showed their absence. Our studies showed a significant decrease of catechin contents in the cookies prepared from ASO with values ranging from 8.49 ± 0.01 mg/kg to 8.39 ± 0.01 mg/kg from baseline to the 60th day of storage with their absence in the cookies prepared from HVF. On the other hand, the caffeic acid contents on analysis were found ranging 7.80 ± 0.02 mg/kg to 7.71 ± 0.01 mg/kg from 0 to 60th days in ASO cookies with a significant decrease while the HVF cookies do not show any active ingredient contents during the entire storage period. Increase in moisture during storage of cookies is associated with different physicochemical changes including oxidative stress, formation of FFAs, chemical reaction between proteins and reducing sugars, and excessive caramelization resulted in the formation of off odors, objectionable aroma, and undulant color of the cookies. TBARS is an important indicator for the quality of stored food (Butt, Arshad, Alam, & Nadeem, 2007; Wada, 1998). Slow increase in moisture of ASO cookies caused the sustainability of total acidity and peroxide value that is directly related to antioxidant potential of ASO cookies.

### 3.4 Sensory evaluation of cookies

Hedonic response is crucial to judge the product for consumer convenience, acceptability, and product feasibility is highly attributed with good sensorial retorts. Before sensory evaluation, training and instructions were given to the all participants so that they can evaluate the products for sensory evaluation in the right way. The mean rating scores of the 9‐point (low to high) sensory evaluation scale of color, flavor, taste, crispness, and overall acceptability are shown in Table 3 which shows that ASO cookies at baseline were superior in evaluation of color, flavor, taste, crispness, and overall acceptability as compared with HVF cookies. The mean evaluation of color in ASO cookies decreased from 8.72 ± 0.02 at baseline to 8.17 ± 0.01 at day 60; on the other hand, same decreasing trend of color evaluation was observed in HVF cookies over time. Similarly, flavor evaluation decreased from baseline 7.72 ± 0.01 to 60th day 6.98 ± 0.01 in ASO cookies and 6.91 ± 0.01 at day 0 to 6.35 ± 0.02 at day 60. On the termination of study, significant (*p* < .05) differences were observed between the groups in different sensory attributes. Different sensory attributes were found ranked higher in ASO cookies as compared to HVF cookies. Both ASO and HVF cookies showed similar physical attributes at all three time intervals as shown in Figure 1. Diameter of HVF cookies significantly (*p* < .05) increased from baseline to day 60, and thickness of both cookies decreased significantly over time, while a similar increasing trend in terms of spread factor was observed in both ASO and HVF cookies. Sensory attributes were negatively affected by the unwanted increase in moisture contents of the cookies during storage that is associated with the disliking of the product due to quality defects. A number of studies showed the same tendency of the drastic effects of upsurge in moisture during storage and an ultimate decline in the quality of the final product which is directly proportional to the poor marketability and reduced acceptability of the products (Waheed et al., 2010). During storage, the percentage of absorbance of moisture increased that result in an increased diameter and a reduced thickness of cookies. Physical properties are also directly related to composition of cookies. As in composition of both cookies, the major variation was the ASO and HVF that creates the differences during storage. There is no prior information available about the utilization of Ajwa date seed oil (ASO) as an active ingredient in human diets; however, usage of date pits in animal feed and as a substitute of plane caffeine free coffee is evident from the literature. Recently, date seed oil was effectively utilized as an alternative source of conventional HVFs by Basuny and Al‐Marzooq (2011), in concocting of mayonnaise that was found superior in the sensory characteristics and quality attributes as compared with that of corn oil. Similarly, Mirghani (2012) experimented with date pits and formulated date pit jam that was also found satisfactory in sensory characteristics. Recently, some researchers have tried to utilize this neglected by‐product for its possible usage including its active constituents in human diet; in this domain, Mirghani (2012) made delicious date pit cordial drink by using date pit powder, sucrose, ascorbic acid, and citric acid. The drink was judged by a panel of 30 experts and was assigned mean overall acceptability of 4.30. Likewise, Salem, Almohmadi, and Al‐Khataby (2011) prepared muffins and an Arabian fermented product called Shabora by the addition of date seed powders at various increments of 2%–10% on weight basis, on their sensory evaluation by a panel of experts reported that the products containing 10% of date seed powders were superior in sensory characteristics than others. Previously, in the preparation of Saudi Mafrood flat breads date seed powder at different rates ranging from 0% to 15% was incorporated, and it was concluded from their results that the breads having 10% date seed powder were similar in almost all attributes on sensory evaluation as compared with the control breads prepared with wheat bran (Almana & Mahmoud, 1994).

**Table 3:** Palatability of functional cookies made from Ajwa seed oil

Characteristics	Day 0	Day 30	Day 60
Color			
ASO	8.72 ± 0.02a	8.43 ± 0.01b	8.17 ± 0.01c
HVF	7.56 ± 0.01d	7.13 ± 0.01e	6.98 ± 0.01f
Flavor			
ASO	7.72 ± 0.01a	7.24 ± 0.01b	6.98 ± 0.01c
HVF	6.91 ± 0.01d	6.64 ± 0.03e	6.35 ± 0.02f
Taste			
ASO	8.24 ± 0.01a	7.29 ± 0.01c	6.91 ± 0.01e
HVF	7.77 ± 0.01b	7.29 ± 0.01c	6.96 ± 0.01d
Texture			
ASO	7.68 ± 0.01a	7.00 ± 0.01b	6.88 ± 0.00d
HVF	6.91 ± 0.01c	6.64 ± 0.02e	6.44 ± 0.01f
Crispness			
ASO	7.58 ± 0.01a	7.22 ± 0.01b	6.99 ± 0.01c
HVF	6.83 ± 0.02d	6.54 ± 0.02e	6.40 ± 0.01f
Overall acceptability			
ASO	8.51 ± 0.01a	7.68 ± 0.01b	7.23 ± 0.02d
HVF	7.26 ± 0.00c	7.00 ± 0.02e	6.86 ± 0.03f

Note

Means showing similar letter(s) in a row/column are nonsignificant (*p* > .05, *n* = 3). Mean ± *SE*.

**Figure 1:** Physical properties of functional cookies made from Ajwa seed oil

## 4 CONCLUSION

Outcomes of this current study showed that the substitution of conventional partially HVF/shortenings or plastic fats with Ajwa date seed oil (ASO) in cookies preparation results in significant improvement in the physicochemical properties, antioxidantal indices, sensory attributes, and physical properties. Over a storage period of 60 days, results revealed that almost all of the properties were found in a decreasing order in both types of cookies including ASO and HVF cookies. Whereas ASO cookies were found more stable in terms of physical properties and acceptability due to the presence of functional moieties that could be a good addition being healthful as a functional food item as compared with the HVF cookies deprived of healthful benefits. Utilization of the antioxidantal potential of Ajwa date seed oil against the drastic effects of oxidation and biochemical reactions that in turn reduce the shelf life of the product could be a better choice for the industries looking for formulating the products like cookies with novel functional properties. By substituting the source of fat with ASO, high standards of nutritional potential with the desired physical properties, improved palatability, and increased shelf life could be achieved by the industries in cookies manufacturing without any additional cost, as the cost of production of both types of cookies was almost the same in addition to the value addition of the discarding material and the proposed health benefits.

## CONFLICT OF INTEREST

The authors have no conflict of interest for this article.

## ETHICAL APPROVAL

This study has nothing to do with human and animal testing.

## References

[fsn31383-bib-0001] AACC (2000). Approved methods of American Association of Cereal Chemists, Inc. AACC: St. Paul, MN.

[fsn31383-bib-0002] Abdul Afiq, M. J. , Abdul Rahman, R. , Che Man, Y. B. , Al‐Kahtani, H. A. , & Mansor, T. S. T. (2013). Date seed and date seed oil. International Food Research Journal, 20(5), 2035–2043.

[fsn31383-bib-0003] Aldhaheri, A. , Alhadrami, G. , Aboalnaga, N. , Wasfi, I. , & Elridi, M. (2004). Chemical composition of date pits and reproductive hormonal status of rats fed date pits. Food Chemistry, 86(1), 93–097. 10.1016/j.foodchem.2003.08.022

[fsn31383-bib-0004] Al‐Farsi, M. A. , & Lee, C. Y. (2008). Nutritional and functional properties of dates: A review. Critical Review in Food Science and Nutrition, 48(10), 877–887. 10.1080/10408390701724264 18949591

[fsn31383-bib-0005] Alfenas, R. C. G. , & Mattes, R. D. (2003). Effect of fat sources on satiety. Obesity Research, 11(2), 183–187. 10.1038/oby.2003.29 12582212

[fsn31383-bib-0006] Almana, H. A. , & Mahmoud, R. M. (1994). Palm date seeds as an alternative source of dietary fiber in Saudi bread. Ecology of Food and Nutrition, 32, 261–270. 10.1080/03670244.1994.9991406

[fsn31383-bib-0007] AOAC (1990). Association of Official Analytical Chemists, official methods of analysis (15th ed.). Washington, DC: Association of Official Analytical Chemists.

[fsn31383-bib-0008] Arshad, H. R. , Salah, M. A. , Habeeb, A. , Babiker, A. Y. , Srikar, S. , & Amjad, A. K. (2014). Therapeutic effects of date fruits (*Phoenix dactylifera* L.) in the prevention of diseases via modulation of anti‐inflammatory, anti‐oxidant and anti‐tumour activity. International Journal of Clinical and Experimental Medicine, 7(3), 483–491.24753740PMC3992385

[fsn31383-bib-0009] Arshad, M. S. , Batool, S. M. , Khan, M. K. , Imran, M. , Ahmad, M. H. , Anjum, F. M. , & Hussain, S. (2019). Bio‐evaluation of functional date bars using rats as model organism against hypercholesterolemia. Lipids in Health and Disease, 18(1), 148 10.1186/s12944-019-1087-3 31272450PMC6610949

[fsn31383-bib-0010] Aslam, F. , Iqbal, S. , Nasir, M. , Anjum, A. A. , Swan, P. , & Sweazea, K. (2018). Effect of hydrogenated fat replacement with white sesame seed oil on physical, chemical and nutritional properties of cookies. Italian Journal of Food Science, 30, 13–025. 10.14674/IJFS-703

[fsn31383-bib-0011] Basuny, A. M. M. , & Al‐Marzooq, M. A. (2011). Production of mayonnaise from date pit oil. Food and Nutrition Sciences, 2, 938–943. 10.4236/fns.2011.29128

[fsn31383-bib-0012] Besbes, S. , Blecker, C. , Deroanne, C. , Bahloul, N. , Lognay, G. , Drira, N. E. , & Attia, H. (2004). Date seed oil: Phenolic, tocopherol and sterol profiles. Journal of Food Lipids, 11(4), 251–265. 10.1111/j.1745-4522.2004.01141.x

[fsn31383-bib-0013] Besbes, S. , Blecker, C. , Deroanne, C. , Drira, N. E. , & Attia, H. (2004). Date seeds: Chemical composition and characteristic profiles of the lipid fraction. Food Chemistry, 84, 577–584. 10.1016/S0308-8146(03)00281-4

[fsn31383-bib-0014] Besbes, S. , Blecker, C. , Deroanne, C. , Lognay, G. , Drira, N. E. , & Attia, H. (2005). Heating effects on some quality characteristics of date seed oil. Food Chemistry, 91, 469–476. 10.1016/j.foodchem.2004.04.037

[fsn31383-bib-0015] Biglar, M. , Khanavi, M. , Hajimahmoodi, M. , Hassani, S. , Moghaddam, G. , Sadeghi, N. , & Oveisi, M. R. (2012). Tocopherol content and fatty acid profile of different Iranian date seed oils. Iranian Journal of Pharmaceutical Research, 11(3), 873–878.24250514PMC3813139

[fsn31383-bib-0016] Blainski, A. , Lopes, G. C. , & De Mello, J. C. P. (2013). Application and analysis of the Folin Ciocalteu Method for the determination of the total phenolic content from (*Limonium brasiliense* L.). Molecules, 18(6), 6852–6865. 10.3390/molecules18066852 23752469PMC6270247

[fsn31383-bib-0017] Butt, M. S. , Arshad, M. U. , Alam, M. S. , & Nadeem, M. T. (2007). Bioavailability and storage stability of vitamin A fortificant (*Retinyl acetate*) in fortified cookies. Food Research International, 40(10), 1212–1219. 10.1016/j.foodres.2007.07.002

[fsn31383-bib-0018] Devshony, S. , Eteshola, A. , & Shani, A. (1992). Characteristics and some potential application of date palm (*Phoenix dectlifera* L.) seeds and seed oil. Journal of American Oil Chemists' Society, 69, 595–597. 10.1007/BF02636115

[fsn31383-bib-0019] Galeb, H. A. , Salimon, J. , Eid, E. E. M. , Nacer, N. E. , Saari, N. , & Saadi, S. (2012). The impact of single and double hydrogen bonds on crystallization and melting regimes of Ajwa and Barni lipids. Food Research International, 48(2), 657–666. 10.1016/j.foodres.2012.06.006

[fsn31383-bib-0020] Garcia‐Alonso, M. , De Pascual‐Teresa, S. , Santos‐Buelga, C. , & Rivas‐Gonzalo, J. C. (2004). Evaluation of the antioxidant properties of fruits. Food Chemistry, 84(1), 13–018. 10.1016/S0308-8146(03)00160-2

[fsn31383-bib-0021] Giarnetti, M. , Paradiso, V. M. , Caponio, F. , Summo, C. , & Pasqualone, A. (2015). Fat replacement in shortbread cookies using an emulsion filled gel based on inulin and extra virgin olive oil. LWT‐Food Science and Technology, 63(1), 339–345. 10.1016/j.lwt.2015.03.063

[fsn31383-bib-0022] Guizani, N. , Suresh, S. , & Rahman, M. S. (2014). Polyphenol contents and thermal characteristics of freeze dried date pits powder Paper presented at the international conference of agricultural engineering, Zurich. 06‐10.07.2014. Ref: C0296: 1‐08. http://www.eurageng.eu

[fsn31383-bib-0023] Hamad, I. , AbdElgawad, H. , Al Jaouni, S. , Zinta, G. , Asard, H. , Hassan, S. , … Selim, S. (2015). Metabolic analysis of various date palm fruit (*Phoenix dactylifera* L.) cultivars from Saudi Arabia to assess their nutritional quality. Molecules, 20(8), 13620–13641. 10.3390/molecules200813620 26225946PMC6331958

[fsn31383-bib-0024] Jayasekera, S. , Molan, A. L. , Garg, M. , & Moughan, P. J. (2011). Variation in antioxidant potential and total polyphenol content of fresh and fully fermented Sri Lankan tea. Food Chemistry, 125(2), 536–541. 10.1016/j.foodchem.2010.09.045

[fsn31383-bib-0025] Jisha, S. , Padmaja, G. , Moorthy, S. N. , & Sajeev, M. S. (2009). Textural and rheological properties of whey protein concentrate fortified baked products from cassava‐based composite flours. Journal of Food Science and Technology Mysore, 46(6), 532–537.

[fsn31383-bib-0026] Kwaasi, A. A. A. (2003). Date palm and sandstorm borne allergens. Journal of Clinical and Experimental Allergy, 33(4), 419–426. 10.1046/j.1365-2222.2003.01635.x 12680855

[fsn31383-bib-0027] Lunn, G. (2000). HPLC methods for pharmaceutical analysis. New York, NY: Interscience Publication.

[fsn31383-bib-0028] Meilgaard, M. C. , Civille, G. V. , & Carr, B. T. (2007). Sensory evaluation techniques (4th ed.). New York, NY: C.R.C. Press L.L.C.

[fsn31383-bib-0029] Mirghani, M. E. S. (2012). Processing of Date Palm Kernel (DPK) for production of nutritious drink. Advances in Natural and Applied Sciences, 6(5), 575–582.

[fsn31383-bib-0030] Mortadha, A. A. , Tahseen, A. A. H. , & Imad, A. A. H. (2015). Extraction of date palm seed oil (*Phoenix dactylifera* L.) by soxhlet apparatus. International Journal of Advances Engineering and Technology, 8(3), 261–271.

[fsn31383-bib-0031] Nagi, H. P. S. , Kaur, J. , Dar, D. , & Sharma, S. (2012). Effect of storage period and packaging on shelf life of cereal bran incorporated cookies. American Journal of Food Technology, 7(5), 301–310. 10.3923/ajft.2012.301.310

[fsn31383-bib-0032] Nanditha, B. , & Prabhasankar, P. (2009). Antioxidant in bakery products: A review. Critical Reviews in Food Science and Nutrition, 49(1), 1–027. 10.1080/10408390701764104 18949596

[fsn31383-bib-0033] Pasha, I. , Butt, M. S. , Anjum, F. M. , & Shehzadi, N. (2002). Effect of dietetic sweeteners on the quality of cookies. International Journal of Agriculture and Biology, 4(2), 245–248.

[fsn31383-bib-0034] Quilez, J. , Ruiz, J. A. , Brufau, G. , & Rafecas, M. (2006). Bakery products enriched with phytosterols, α‐tocopherol and β‐carotene. Sensory evaluation and chemical comparison with market products. Food Chemistry, 94(3), 399–405. 10.1016/j.foodchem.2004.11.029

[fsn31383-bib-0035] Rahman, M. S. , Kasapis, S. , Al‐Kharusi, N. S. Z. , Al‐Marhubi, I. M. , & Khan, A. J. (2007). Composition characterization and thermal transition of date pits powders. Journal of Food Engineering, 80(1), 1–10. 10.1016/j.jfoodeng.2006.04.030

[fsn31383-bib-0036] Rangrej, V. , Shah, V. , Patel, J. , & Ganorkar, P. (2015). Effect of shortening replacement with flaxseed oil on physical, sensory, fatty acid and storage characteristics of cookies. Journal of Food Science and Technology, 52(6), 3694–3700. https://doi.org/10.1007%252Fs13197-014-1430-7 2602875310.1007/s13197-014-1430-7PMC4444888

[fsn31383-bib-0037] Reddy, V. , Urooj, A. , & Kumar, A. (2005). Evaluation of antioxidant activity of some plant extracts and their application in biscuits. Food Chemistry, 90(1–2), 317–321. 10.1016/j.foodchem.2004.05.038

[fsn31383-bib-0038] Salem, E. M. , Almohmadi, N. , & Al‐Khataby, N. F. (2011). Utilization of Date seeds powder as antioxidant activities components in preparation of some baking products. Journal of Food and Dairy Science, 2, 399–409.

[fsn31383-bib-0039] Sharif, K. , Butt, M. S. , Anjum, F. M. , Nasir, M. , Minhas, R. , & Qayyum, M. M. N. (2003). Extension of cookies shelf life by using rice bran oil. International Journal of Agriculture and Biology, 5(4), 455–457.

[fsn31383-bib-0040] Steel, R. G. D. , Torrie, J. H. , & Dickey, D. A. (1997). Principles and procedures of statistics: A biometrical approach (3rd ed., pp. 352–358). New York, NY: McGraw Hill Book Co., Inc.

[fsn31383-bib-0041] Sumaira, K. , Nauman, K. , Rao Sanaullah, K. , Haroon, A. , & Asif, A. (2017). A review on chemistry and pharmacology of Ajwa date fruit and pit. Trends in Food Science and Technology, 63, 60–69. 10.1016/j.tifs.2017.02.009

[fsn31383-bib-0042] Wada, P. (1998). Biscuits, cookies and crackers: The principle of the craft (1st ed.). London, UK: Elsevier Applied Science.

[fsn31383-bib-0043] Waheed, A. , Rasool, G. , & Asghar, A. (2010). Effect of interesterified palm and cotton seed oil blends on cookie quality. Agriculture and Biology Journal of North America, 1(3), 402–406. 10.5251/abjna.2010.1.3.402.406

[fsn31383-bib-0044] Wang, F. C. , Gravelle, A. J. , Blake, A. I. , & Marangoni, A. G. (2016). Novel trans‐fat replacement strategies. Current Opinion in Food Science, 7, 27–34. 10.1016/j.cofs.2015.08.006

[fsn31383-bib-0045] Xin, M. , Yuan, W. , Xiao, W. , & You‐Ying, T. (2011). Antagonism of phenanthrene cytotoxicity for human embryo lung fibroblast cell line HFL‐I by green tea polyphenol. Environmental Pollution, 159(1), 164–168. 10.1016/j.envpol.2010.09.010 20932619

